The article "Phenotypic Changes of LncRNA Hotair in Non-Small-Cell Lung Cancer and Its Clinical Application" was retracted in 2023. Reasons: unreliable results or conclusions; concerns about the data; concerns about the peer review; concerns about the citations.

# Phenotypic Changes of LncRNA Hotair in Non-Small-Cell Lung Cancer and Its Clinical Application

**DOI:** 10.1155/2021/3215143

**Published:** 2021-11-05

**Authors:** Haihua Huang, Jin Wang, Fabing Liu

**Affiliations:** ^1^Department of Thoracic Surgery Shanghai General Hospital, Shanghai Jiao Tong University School of Medicine, 100Haining Road, Shanghai 200080, China; ^2^Department of Thoracic Surgery, Shanghai East Hospital, Tongji University, School of Medicine, Shanghai 200120, China

## Abstract

Non-small-cell lung cancer (NSCLC) is one of the main causes of death of malignant tumors of the respiratory system. At present, the clinical demand for biomarkers for predicting and diagnosing the disease is increasing. Overexpression of LncRNA Hotair (Homeobox transcriptional antisense intergenic RNA) has been previously reported to be associated with poor prognosis and high mortality in different malignancies. qRT-PCR results showed that the expression of LncRNA Hotair in tumor tissue and serum of patients with non-small-cell lung cancer was significantly upregulated. Clinicopathological correlation analysis showed that the upregulation of LncRNA Hotair expression was closely related to lymph node metastasis and tumor lymph node metastasis (TNM) stage (*P* < 0.05). The results showed that transfection of pcDNA3.1-Hotair could promote the expression of LncRNA Hotair in NSCLC, while transfection of Si-Hotair could reduce the expression level of LncRNA Hotair, hinder the migration and invasion of cancer cells, and promote cell apoptosis. After transfection of Si-Hotair, molecular markers related to migration, the level of E-cadherin and Bax, increased and the level of vimentin, Bcl-2, MMP-3, VEGF, Ki-67 and PCNA decreased. This shows that the proliferation and migration of A549 cells are promoted and LncRNA Hotair deletion can inhibit the proliferation and migration of lung cancer cells. These results show that the expression level of LncRNA Hotair of NSCLC cell lines can promote the invasion and migration of NSCLC, and its expression has a significant correlation with Lymph node metastasis, tumor size, and TNM stage. Therefore, this target is of great significance for the clinical diagnosis and treatment of NSCLC.

## 1. Introduction

Non-small-cell lung cancer (NSCLC) is one of the most common malignant tumors of the respiratory system. The main causes of death are smoking, low air quality, gene mutation, and other adverse factors, and its new cases in the world are increasing year by year, especially in China [1, 2]. Although some progress has been made in clinical and experimental research, the long-term prognosis of NSCLC patients is still very poor due to late discovery of the disease, high recurrence rate, and lack of an effective treatment intervention for advanced tumors. Previous studies have revealed many dysregulated genes and signaling pathways associated with NSCLC, but the highly complex molecular mechanism of its carcinogenesis and progression is still unclear [3]. Therefore, it is urgent to find reliable biomarkers for early diagnosis, effective treatment, and prognosis evaluation of NSCLC.

Long non-coding RNA (LncRNA) is a subcategory of the nontranslated RNA sequence defined by more than 200 base pairs of any length [4, 5]. Studies have found the physical location and protein coding of most LncRNAs. The genes are very close, and they can be further classified according to the order of coding and the positional relationship. They are divided into intergenic LncRNA, antisense LncRNA, and other subtypes [6, 7].The change of LncRNA content in plasma, serum, or urine has become an emerging technology for noninvasive diagnostic applications [8, 9]. For example, plasma LncRNA-Pou3f3 can be used as a potential biomarker for the diagnosis of rectal cancer, especially early tumor screening [10]. LncRNA Loc389332 was found to be significantly increased in the plasma and urine of patients with renal clear cell carcinoma, which can be used to distinguish cancer patients from the health examination group [11]. LncRNA Hotair is composed of 2158 nucleotides, located between Hoxc11 and Hoxc12 on chromosome 12q13.135 [12]. It can bind to PRC2, resulting in histone methylation and transcriptional silencing [13]. Studies have shown that, in oral squamous cell carcinoma, LncRNA Hotair overexpression enhances the metastatic potential and epithelial mesenchymal transformation characteristics of cancer cells. It is also found that LncRNA Hotair expression is positively correlated with mesenchymal markers and negatively correlated with epithelial markers in clinical samples [14, 15]. In addition, LncRNA Hotair can realize its function by reprogramming the chromosome state to control the expression of multiple genes represented by Hoxc10; Hoxc10 has been proved to be a gene closely related to tumor pathogenesis, and its expression is also significantly increased in cancer tissues of individuals with lymph node metastasis [16].

Based on the conclusions of previous studies, this paper further studied the relationship between the expression level and pathological parameters of LncRNA Hotair in clinical samples of NSCLC and the related mechanism of exogenous LncRNA Hotair on cell proliferation, migration, and invasion, so as to fully grasp the role of LncRNA Hotair in NSCLC. It provides valuable clinical auxiliary reference for the treatment of NSCLC.

## 2. Materials and Methods

### 2.1. Patient Samples and Materials

During the research process, 62 patients with NSCLC in the hospital from January 2018 to December 2020 were selected from cancer tissues and adjacent paracancerous tissue specimens. In the course of the study, all patients had not received chemotherapy or targeted therapy before surgery and signed an agreement to participate in the experiment with the patients. This study was approved by the ethics committee of Shanghai General Hospital, Shanghai Jiao Tong University, School of Medicine. Clinical data including age, sex, smoking history, stage, and lymph node metastasis of these patients were collected. All specimens were placed in liquid nitrogen for cryopreservation after sampling. The lung cancer cells used can be divided into an adenocarcinoma cell line (A549, SPC-A1), squamous cell carcinoma cell line (SK-MES-1), and human normal bronchial epithelial cell line, and they were purchased from the Institute of Biochemistry and Cell Biology, Chinese Academy of Sciences, Shanghai, China. RPMI 1640 medium, DMEM medium, 10% fetal bovine serum, Trizol reagent, plasmid expression vector pc3.1DNA, three independent small interfering RNAs (siRNAs), negative control siRNA (si-NC), and transfection reagent were purchased from Invitrogen company of the United States; the PrimeScript reverse transcription kit and SYBR Premix Ex Taq were purchased from Shanghai Shenggong company.

### 2.2. Cell Culture

In the experiment, DMEM medium, RPMI1640 medium, fetal bovine serum (10%), and cell culture medium were used for sample cell culture, and 10% fetal bovine serum, penicillin, and streptomycin were added to the culture medium. The cells of the small cell lung cancer tissue sample were cultured at 37 degrees Celsius and 5% CO2. In order to construct LncRNA Hotair expression vector, a full-length Hotair fragment was amplified from the cDNA of NSCLC cells by PCR. The PCR product was verified and subcloned into mammalian expression vector pc3.1DNA.

### 2.3. Cell Transfection

NSCLC cells in the logarithmic growth stage were inoculated into 6-well plates 24 hours before transfection and transfected when the cell growth fusion degree reached 70%–80%. We transfected pcDNA3.1-Hotair into NSCLC cells and control antagomirs (anti-NC) and si-Hotair into NCSCLC cells. After the transfection was completed, we continued to culture and set a blank vector and a negative control group (Si-NC) cultivated together, and the culture period is 2 days. Cells from each group were collected 48 hours after transfection for qRT-PCR analysis.

### 2.4. Quantitative Real-Time RT-PCR

Extract PCR for reverse transcription used PrimeScript and SYBR Premix Ex Taq reagents as transcription reagents to detect the transcription efficiency, and quantitative detection and data recording of its transfection rate were performed. LncRNA Hotair upstream primer: 5′-TAGGCAAATGTCAGGTT-3′ and downstream primer: 5′-ACACAAGTAGCAGGAAAGG-3′. GAPDH primer upstream primer: 5′-CGAG ATCCCTCCAAAATCAA-3′ and downstream primer: 5′-wTTCACACCCATGAC GAACAT-3′.

### 2.5. Cell Counting Kit-8 (CCK-8) Assay

Cell proliferation assay was performed with CCK-8 assay according to the manufacturer's protocol. The cells were seeded into 96-well plates with 1 × 10^4^ cells per well in triplicate. CCK-8 (10 *μ*L) was added to each well at different time points (0, 1, 2, 3, 4, and 5 days) and then incubated in the dark for 2 h at room temperature. The absorbance was measured at 450 nm using a microplate spectrophotometer.

### 2.6. Cell Migration and Invasion Experiment

Transwell experiment was performed 48 hours after transfection. In the migration experiment, 5 × 10^4^ cells were added to the upper serum-free medium; in the invasion experiment, 1 × 10^5^ cells were added to the upper serum-free medium; the lower chamber was a medium containing 10% fetal bovine serum. After incubation for 24 hours, the cells migrated or invaded to the lower layer were fixed with methanol, stained with 0.1% crystal violet, and counted with an inverted microscope. The experiment was repeated three times independently.

### 2.7. DAPI Staining Was Used to Observe the Morphological Changes of SPC-A1 Cell Apoptosis

SPC-A1 cells were cultured in a 37°C incubator for 48 hours; then, the culture was terminated, washed with PBS for 3 times, then fixed with 4% paraformaldehyde for 5 min, diluted with a DAPI dye solution to make its final concentration 50 *µ*mol/L, 100 *µ*L per well, and stained at room temperature without light for 20 min. After washing with PBS, the morphological changes of cells in each group were observed under a fluorescence microscope.

### 2.8. Apoptosis Was Detected by TUNEL and Merge Staining

SPC-A1 cells in the logarithmic growth stage were treated with 1 × 10^8^/L and inoculated into 96-well plates, 100 *µ*L per well, cultured in a 37°C incubator for 24 hours, and the culture was terminated after the cells adhered to the wall and continued to be cultured at 37°C for 48 hours, 4% paraformaldehyde was fixed for 30 min and then cleaned twice with PBS, equilibrium buffer was added and incubated at room temperature for 5 min, finally 50 *µ*L reaction buffer was added, incubated in the dark for 60 min, and centrifuged with a centrifuge, the supernatant was discarded and 5xWash with 10-3 mg/L BSA was added, and the morphological changes of cells were observed under a fluorescence microscope and photos were taken.

### 2.9. Western Blot

The total protein of cells in each group after 48 hours of transfection was extracted and quantified according to each 1 *μ*L sample added 0.25 *μ*L. The ratio of sample buffer was mixed, boiling water heating denatured 5 min, separated by SDS-PAGE gel electrophoresis, and migrated to a nitrocellulose membrane, and 5 g defatted milk powder and 100 mL TBST closed buffer were added and placed in an oscillating incubator at 26°C closed for 2 h. The primary antibodies used in this study include Ki-67, proliferating cell nuclear antigen (PCNA), Bax, Bcl-2, matrix metalloproteinase-3 (MMP-3), vascular endothelial growth factor (VEGF), epithelial cadherin (E-cadherin), vimentin, and GAPDH. The membranes were then incubated with horseradish peroxidase-conjugated goat anti-rabbit or goat anti-mouse secondary antibody for 1 h at room temperature. Then, the antibody-bound proteins were detected using the ECL system.

### 2.10. Statistical Analysis

After completing the experiment, based on the quantitative detection and recorded experimental data, all statistical analyses were performed using SPSS software package version 22.0 (SPSS, Chicago, Illinois, USA). All graphics were drawn by Graphpad prism 9.0 software (GraphPad software, La Jola, California). A paired-sample *t*-test was used to compare the difference of Hotair expression in paired tissues of NSCLC patients. Other experimental data were compared by an independent *t*-test; ^*∗*^ represents <0.05, ^*∗∗*^ represents <0.01, and ^*∗∗∗*^ represents <0.001.

## 3. Results

### 3.1. Higher Expression of LncRNA Hotair in NSCLC Tissue

In order to investigate the expression of LncRNA Hotair in NSCLC patients, we first performed qRT-PCR to determine the expression level of LncRNA Hotair in NSCLC and adjacent tissues. In the independent study group of 62 original NSCLC patients, the expression level of LncRNA Hotair was (25.30 ± 2.23) in NSCLC tissues and (3.52 ± 0.29) in adjacent tissues (Figure 1). The expression level of LncRNA Hotair was significantly higher than that of adjacent tissues (*P* < 0.0001).

### 3.2. Correlation between Clinicopathological Parameters and Relative Expression of LncRNA Hotair

In order to further study the role of LncRNA Hotair in the occurrence and development of NSCLC, this study statistically analyzed the relationship between serum LncRNA Hotair level and clinicopathological parameters in patients with NSCLC. The results showed that there was no significant correlation between serum LncRNA Hotair level and gender, age, and smoking (*P* > 0.05). The serum LncRNA Hotair level of lung cancer patients with tumor size >3 cm was significantly higher than that of patients with tumor size ≤3 cm, the serum LncRNA Hotair level of patients with stage III + IV NSCLC was significantly higher than that of patients with stage I + II, and the serum LncRNA Hotair level of NSCLC patients with lymphatic metastasis was significantly higher than that of patients without lymphatic metastasis (*P* < 0.001). The results are shown in Table 1.

### 3.3. Expression Level of Exogenous LncRNA Hotair in NSCLC Cells and Changes in Silencing and Overexpression Levels

The expression content of LncRNA Hotair in NSCLC tissues was higher than that in adjacent tissues. It can be seen from the table that the relative expression value of SPC-A1 and SK-MES-1 cell lines is higher than that of normal cell lines, and the relative expression value of A549 cell line is lower than that of normal cell lines, as shown in Figure 2(a). In order to further verify the correlation between the expression level of LncRNA Hotair, the expression level of exogenous LncRNA Hotair in NSCLC cells was observed by transfection and overexpression, and an A549 cell line with the lowest expression and an SPC-A1 cell line with the highest expression were selected for verification. Also, from the histogram of the relative expression level, the relative expression level showed an obvious difference, which was more obvious in the Hotair group. Based on the abovementioned analysis, it can be clearly seen that, after 2 days of transfection with siRNA, the expression level of LncRNA Hotair in SK-MES-1 and SPC-A1 cells was lower than before transfection (*P* < 0.05). RNA interference technology can inhibit the proliferation of NSCLC cells by hindering the expression level of LncRNA Hotair. Transfection of pcDNA3.1-Hotair promoted the expression of Hotair and inhibited the proliferation of NSCLC cells. After 2 days of transfection with pcDNA3.1-Hotair, the expression level of LncRNA Hotair in SK-MES-1 and SPC-A1 cells was higher than before transfection (Figures 2(b) and 2(c)).

### 3.4. Downregulation of LncRNA Hotair Suppressed Cell Proliferation and Invasion and Promoted Apoptosis of NSCLC Cells

In order to study the role of LncRNA Hotair in NSCLC, siRNA was used to specifically downregulate the expression of LncRNA Hotair. Because the expression of LncRNA Hotair in SPC-A1 and sK-MES-1 cell lines was higher, we chose the SPC-A1 cell line for the next experiment.We found that compared with NC and anti-NC groups, LncRNA Hotair downregulated inhibited cell proliferation and promoted apoptosis, and DAPI staining showed that the tumor cells in the Si-Hotair group and Si-Hotair + anti-NC group showed shrinkage, dense cytoplasm, edge collection of nuclear chromatin, nuclear lysis, and formation of apoptotic bodies containing nuclear fragments and organelles. The downregulation of LncRNA Hotair suppressed cell proliferation (Figure 3(a)). TUNEL and Merge staining showed that the proportion of green fluorescence positive cells in the Si-Hotair group and Si-Hotair + anti-NC group increased gradually, indicating that the proportion of apoptosis increased gradually (Figures 3(b) and 3(c)). Si-Hotair also inhibited the invasive ability of SPC-A1 cells (Figures 3(d) and 3(e)). Si-Hotair decreased the expression of proliferation-related proteins Ki-67 and proliferating cell nuclear antigen (PCNA), E-cadherin and vimentin, anti-apoptotic protein Bcl-2, and invasion-related protein matrix metalloproteinase-3(MMP-3) and vascular endothelial growth factor (VEGF), while the expression of proapoptotic protein Bax increased significantly (Figures 4(a)–4(c)). In addition, the expression of epithelial marker E-cadherin was upregulated, while the expression of mesenchymal marker vimentin was downregulated. Si-Hotair could inhibit epithelial mesenchymal like phenotypic transformation (EMT) in NSCLC (Figure 4(d)). In conclusion, our results showed that the downregulation of LncRNA Hotair inhibited cell proliferation and invasion and promoted the apoptosis of NSCLC cells.

## 4. Discussion

Lung cancer is the leading cause of cancer-related death, and NSCLC accounts for 85% of all lung cancer patients. In recent years, with the development of molecular biology of lung cancer, many new drugs have appeared, but the 5-year survival rate of patients with advanced lung cancer is still only 15% [17]. In recent years, it has been found that the abnormal expression of lncRNA is closely related to human diseases and is involved in the process of tumor occurrence, growth, invasion, metastasis, recurrence, and drug resistance [18–20].

LncRNA Hotair is the transcriptional antisense RNA of HOX. It is the first LncRNA recognized to have transcriptional regulation and related to malignant tumors. Studies have shown that LncRNA Hotair mainly interacts with Polycomb repressive complex 2 (PRC2) to regulate chromosome rearrangement and promote tumorigenesis[21]. Duan, et al. Found that LncRNA Hotair was highly expressed in liver cancer tissues and promoted hepatocarcinogenesis by inhibiting the expression of tumor suppressor genes; conversely, downregulating LncRNA Hotair expression can inhibit the growth and migration of hepatoma cells [22]. It was found that the overexpression of Hotair in gastric cancer can promote lymph node metastasis, EMT progression, and vascular invasion of gastric cancer [23]. The overexpression of LncRNA Hotair is the main marker of poor prognosis in patients with gastric cancer. In human glioma, LncRNA Hotair can affect the progression of glioma by affecting the expression of inflammatory factors and VEGF [24]. Therefore, LncRNA Hotair explored the biological behavior and possible mechanism of NSCLC cells. The results showed that LncRNA Hotair was abnormally highly expressed in NSCLC cell lines; transfection knockdown of LncRNA Hotair expression significantly inhibited the proliferation, migration, and invasion of NSCLC cells. It is suggested that LncRNA Hotair has the role of oncogene and can promote the proliferation, migration, and invasion of cancer cells.

From the experimental results, it can be seen that the relative expression level of LncRNA Hotair in SPC-A1 and SK-MES-1 cells is higher than that in normal bronchial epithelial cells (*P* < 0.05); the relative expression level in A549 cells was lower than in normal bronchial epithelial cells (*P* < 0.05). After 2 days of transfection with siRNA, the expression level of LncRNA Hotair in A549 and SPC-A1 cells was lower than before transfection (*P* < 0.05). DAPI/TUNEL/Merge experiment showed that Si-Hotair could gradually increase the proportion of apoptosis. At the same time, through cell proliferation comparison experiments, it was found that, after 2 days of transfection with pcDNA3.1-Hotair, the expression level of LncRNA Hotair in A549 cells was higher than before transfection (*P* < 0.05). Transfection of pcDNA3.1-Hotair to promote the expression of Hotair can inhibit the proliferation of NSCLC cells. On this basis, we conducted a series of studies on the phenotypic changes of NSCLC regulated by LncRNA Hotair. Compared with the Si-NC group and NC group, the number of invasion and migration of SPC-A1 cells in Si-Hotair group decreased significantly, and Si-Hotair decreased the expression of proliferation-related proteins (Ki-67 and PCNA), anti-apoptotic protein Bcl-2, and invasion-related proteins (MMP-3 and VEGF), while the expression of proapoptotic protein Bax increased significantly. We found that the expression of E-cadherin was upregulated and vimentin was downregulated and then speculated that Si-Hotair inhibited the development of EMT. Therefore, a series of experimental results show that Si-Hotair can inhibit tumor occurrence and metastasis by regulating the content expression in NSCLC cells. In conclusion, the experimental results show that LncRNA Hotair has a certain impact on the proliferation, migration, and apoptosis of NSCLC tissues and cells, which has a very important reference value for the treatment and early detection of NSCLC.

## Figures and Tables

**Figure 1:** LncRNA Hotair expression was significantly increased in human NSCLC tissues compared to normal lung tissues.

**Figure 2:** Expression level of exogenous LncRNA Hotair in NSCLC cells and changes in silencing and overexpression levels. (a) Relative expression values of LncRNA Hotair in different cell lines; (b) expression of LncRNA Hotair after transfection; and (c) expression of pcDNA3.1-Hotair after transfection.

**Figure 3:** Downregulation of Hotair suppressed cell proliferation and invasion, while it promoted apoptosis of NSCLC cells. SPC-A1 cells were transfected with anti-NC, Si-Hotair, or Si-Hotair + anti-NC. (a) Cell proliferation was determined by the cell counting kit-8 (CCK-8) assay. (b-c) Cell apoptosis was detected by flow cytometric analysis. (d-e) Invasion ability of cells was compared using the Transwell model. The bars show means ± SD of three independent experiments. ^*∗*^*P* < 0.05, ^*∗∗*^*P* < 0.01, and ^*∗∗∗*^*P* < 0.001, compared with the NC and anti-NC group.

**Figure 4:** Relative protein levels of proliferation-related proteins were detected through western blot. (a) Relative protein levels of proteins MMP-3 and VEGF; (b) relative protein levels of proteins Ki-67 and PCNA; (c) relative protein levels of proteins Bax and Bcl-2; and (d) relative protein levels of proteins E-cadherin and vimentin.

**Table 1:** Relationship between clinicopathological parameters and serum Hotair level in NSCLC.

Clinical pathological parameters	Cases (*n*)	Relative expression of Hotair (mean ± SD)	*t*	*P*
Age (yr)			1.901	0.061
>65	21	2.87 ± 0.74		
≤65	41	3.27 ± 0.79		
Gender			0.528	0.600
Male	28	2.81 ± 0.72		
Female	34	2.91 ± 0.70		
Smoking			0.194	0.847
Yes	29	3.17 ± 0.84		
No	33	3.21 ± 0.65		
Tumor size			4.685	<0.001
>3 cm	37	2.98 ± 0.82		
≤3 cm	25	2.20 ± 0.11		
TNM stage			4.280	<0.001
I + II	33	2.86 ± 0.64		
III + IV	29	2.31 ± 0.25		
Lymph node metastasis			7.308	<0.001
Negative	30	3.32 ± 0.47		
Positive	32	2.60 ± 0.29		

## Data Availability

The simulation experiment data used to support the findings of this study are available from the corresponding author upon request.
